RETRACTED

# Using Big Data-Based Neural Network Parallel Optimization Algorithm in Sports Fatigue Warning

**DOI:** 10.1155/2021/2747940

**Published:** 2021-07-14

**Authors:** Yudong Sun, Yahui He

**Affiliations:** School of Physical Education, Fuyang Normal University, Fuyang 236000, China

## Abstract

In high-paced and efficient life and work, fatigue is one of the important factors that cause accidents such as traffic and medical accidents. This study designs a feature map-based pruning strategy (PFM), which effectively reduces redundant parameters and reduces the time and space complexity of parallelized deep convolutional neural network (DCNN) training; a correction is proposed in the Map stage. The secant conjugate gradient method (CGMSE) realizes the fast convergence of the conjugate gradient method and improves the convergence speed of the network; in the Reduce stage, a load balancing strategy to control the load rate (LBRLA) is proposed to achieve fast and uniform data grouping to ensure the parallelization performance of the parallel system. Finally, the related fatigue algorithm's research and simulation based on the human eye are carried out on the PC. The human face and eye area are detected from the video image collected using the USB camera, and the frame difference method and the position information of the human eye on the face are used. To track the human eye area, extract the relevant human eye fatigue characteristics, combine the blink frequency, closed eye duration, PERCLOS, and other human eye fatigue determination mechanisms to determine the fatigue state, and test and verify the designed platform and algorithm through experiments. This system is designed to enable people who doze off, such as drivers, to discover their state in time through the system and reduce the possibility of accidents due to fatigue.

## 1. Introduction

With the rapid development of social economy, in today's fast-paced and efficient life and work, fatal accidents often occur. Especially in the field of road traffic, after a period of driving, the driver will experience fatigue states such as inattention, closed eyes for a long time, and dozing, resulting in a decrease in the driver's perception and judgment of the surrounding environment [1]. The reaction becomes slow and traffic accidents are prone to occur. Moreover, high-speed traffic accidents are often fatal and devastating. According to the traffic accident statistics yearbook, about 30% of road traffic accidents in the year are related to fatigue driving, and the death toll caused by fatigue driving can account for more than 10% of the total number of traffic accident deaths [2]. How to prevent fatigue and reduce accidents caused by fatigue, especially the occurrence of road traffic accidents, has become a major problem for social public safety. If a real-time detection system can be provided in the car, an alarm can be triggered when the driver just appears fatigued, so that the driver can slow down or stop for a rest, and accidents can be avoided. In this case, the development of a high-performance fatigue warning system has become a hot spot in today's society and has attracted increasing attention.

RETRACTED

With the rapid development of Internet technology and the advent of the era of big data, compared with traditional data, big data has 4 V characteristics, namely, massive (volume), rapid change (velocity), multimodality (variety), and value [3]. The 4 V characteristics make it difficult for traditional classification algorithms and processing platforms to process big data. In recent years, the development of parallelization technology and feature selection classification algorithms provides a new perspective for big data processing. DCNN is one of the classification algorithms [4]. An important type of algorithm, which has powerful feature selection ability, generalization ability, and function approximation ability, is widely used in image analysis, speech recognition, target detection, semantic segmentation, face recognition, automatic driving, and other fields. Therefore, based on big data, DCNN research has become a research hot spot of classification algorithms. Although deep learning technology represented by DCNN has made many important breakthroughs in the field of big data classification in recent years, how to reduce network training time and space complexity is still an important issue. In order to overcome the difficulties encountered in DCNN training, researchers have designed many frameworks to process millions of data, such as AlexNet, VGG, ResNet, and Inception series. Among them, AlexNet has 61 million parameters and VGG16 has 138 million parameters; ResNet and Inception V2 contain 1.7 million parameters and 11.26 million parameters, respectively [5]. Such a large number of parameters require huge time cost and hardware resources, and these problems are usually caused by redundant parameters in DCNN; parameter pruning is an effective method to reduce redundant parameters. Not only is it easy to balance the compression rate and performance loss and is compatible with other types of compression methods, but also it has the potential to prevent overfitting, so it has received widespread attention.

This paper designs a feature map-based pruning strategy (PFM), which effectively reduces redundant parameters and reduces the time and space complexity of DCNN training; in the Map stage, the conjugate gradient method (CGMSE) with modified secant lines is proposed. The fast convergence of the conjugate gradient method improves the convergence speed of the network; in the Reduce phase, a load balancing strategy (LBRLA) is proposed to control the load rate, which realizes fast and uniform data grouping, thereby ensuring the parallelization performance of the parallel system. Finally, the related fatigue algorithm's research and simulation based on the human eye are carried out on the PC. The human face and eye area are detected from the video image collected by the USB camera, and the frame difference method and the position information of the human eye on the face are used. To track the human eye area, extract the relevant human eye fatigue characteristics, combine the blink frequency, closed eye duration, PERCLOS, and other human eye fatigue determination mechanisms to determine the fatigue state, and test and verify the designed platform and algorithm through experiments.

RETRACTED

## 2. Related Works

Hammou et al. [6] took advantage of the complementarity of pruning and quantization and reduced the redundant parameters of DCNN to a certain extent through the compression learning of parallel cropping and quantization, but this method does not consider the difference between DCNN layers. Therefore, Yao et al. [7] integrated two different structured sparse regularizations into the original filtering and pruning objective function, which can deceptively perform pruning. However, the pruning efficiency of this algorithm is low. In summary, how to design a reasonable and effective redundant parameter pruning strategy is still a hot issue in the DCNN community.

From a historical perspective, fatigue warning has been widely used in many aspects, such as car driving. In fact, fatigue driving has aroused great interest of scientists a long time ago, and many scholars have proposed and designed corresponding solutions from different perspectives, for example, from the perspectives of medicine, machinery, and computer vision. However, as of today, due to various constraints, a perfect solution to prevent fatigue in all aspects has not yet appeared. At present, it is a more mature and reliable solution to use physiological signal measurement and analysis to determine whether the driver's mental state is fatigued and to make real-time warnings [8]. However, the limitation of this method is also quite obvious; that is, the subject needs to wear the relevant physiological detection sensing equipment for long-term driving or work, which will cause the subject's discomfort and further affect their normal operation. Therefore, fatigue detection and early warning by means of excluding physiological measurements are the focus of the current research.

RETRACTED

As for the security alert of the perimeter, it is mainly realized through intelligent real-time video surveillance, and the detection and recognition of moving targets are mainly involved here. At present, among the research topics included in computer vision, digital image processing, and pattern recognition, the most popular are the detection and recognition of moving targets. The main idea is to classify moving targets in videos through computer vision technology and at the same time where content and status of its movement are described and identified. From the current point of view, this topic has good application prospects in the fields of human-computer interaction, intelligent monitoring, and behavior recognition and analysis [9]. Because of the change in the shape of the target to be detected, its detection accuracy is not high, which is a big difficulty in this subject, because, in the process of video shooting, they are very susceptible to external objective factors such as illumination and partial occlusion. In addition, there may be situations where similar target objects are quite different in shape, while different types of target objects are very close in shape, all of which cause great difficulties in the detection and recognition of moving targets. Although reducing redundant parameters can reduce the time complexity of the algorithm to a certain extent, the impact of the convergence speed of the parameter update algorithm on the DCNN training time cannot be ignored. Because the convergence speed of the stochastic gradient descent method is too slow in the big data environment, there are some algorithms to speed up the convergence. Scholars proposed updating the parameters using the conjugate gradient method. Sohrabi et al. [10] proposed the conjugate gradient method of the nonlinear center of gravity, which satisfies the sufficient descent condition, but only under the Wolfe criterion can the global convergence be guaranteed. Therefore, Wang et al. [11] proposed an unconstrained spectral conjugate gradient method, which improves the search efficiency of the algorithm to a certain extent by modifying the learning step length and conjugate direction of the conjugate gradient method. In addition, Zhou et al. [12] improved the secant condition and accelerated the convergence speed of the conjugate gradient method, but the spectral conjugate gradient method and the secant formula improved conjugate gradient method cannot guarantee the generation of the descending direction. It is necessary for analysis and implementation. Restart to ensure convergence, so the time complexity of the algorithm may be very high. Therefore, looking for a conjugate gradient method that can quickly converge is one of the important issues in the current research.

RETRACTED

The factors that affect the training efficiency of the parallel DCNN algorithm in a big data environment are the convergence speed of the gradient descent method and the performance of the parallel model. In recent years, researchers have proposed many big data processing methods that can effectively improve the efficiency of the algorithm. Among them, the MapReduce parallel developed by Google is favored by scholars and enterprises due to its simple operation, automatic fault tolerance, load balancing, and strong scalability. At present, many neural network algorithms based on the MapReduce calculation model have been successfully applied to the field of big data analysis and processing. Adil et al. [13] proposed the CNN-MR (convolution neural network based MapReduce) algorithm, which uses a data parallel strategy to divide the training samples into each computing node in the platform, which improves the efficiency of algorithm training. Hao et al. [14] proposed DCNN parallel algorithm MR-DCNN (MapReduce based deep convolution neural network algorithm), which reduces the computational complexity of DCNN, but the accuracy of the algorithm is still insufficient. Bhardwaj et al. [15] proposed the PPNN (polymorphic parallel convolution neural network) algorithm, which introduced a deconvolution layer, and improved the accuracy of the algorithm to a certain extent through local polymorphic parallel networks and many-to-many connections. Lakshmanaprabu et al. [16] proposed the DCNN-ABC (deep convolution neural network based parallel artificial bee colony) algorithm, which combines the bee colony algorithm to find the optimal parameters in parallel, and further improved the accuracy of the algorithm. However, the parallel strategy of the above algorithm does not consider the load capacity of the server, resulting in low system operation efficiency and low resource utilization. Therefore, how to design and implement a high-efficiency parallel DCNN is still a problem to be solved.

## 3. Neural Network Parallel Optimization Algorithm Based on Big Data

This article mainly studies the design of an ideal driver fatigue warning system, which requires good real-time performance, low cost, high reliability, all-weather, and intelligence. The system mainly collects the video image of the driver through the camera and uses machine vision technology, image processing technology, face and eye recognition technology, and related fatigue determination algorithms to detect the fatigue state and give an early warning:

1. The Camera Acquires the Image
2. It mainly uses a suitable camera to collect the driver's facial image in real time, mainly including the human face and its background image. In order to make the fatigue warning work normally at night, you can choose a camera with infrared function [17].
3. Image Data Processing
4. In the process of video image acquisition, it may be affected by the interference of external environmental noise and uneven illumination, which leads to the degradation of image quality. In order not to affect the subsequent fatigue feature extraction, it is necessary to perform illumination compensation and image enhancement on the original image to improve the image quality. Then, using related image processing algorithms, we obtain the target area of interest, the human eye area, which provides a basis for subsequent fatigue feature extraction.
5. Feature Extraction of Fatigue State
6. It mainly uses the fatigue determination algorithm to extract the relevant fatigue features from the video image. This article uses the characteristics of the eyes to reflect the fatigue state of the driver. It is necessary to process the face and eyes according to the acquired images to obtain the fatigue characteristics of the eyes, such as the frequency of blinking, the length of time the eyes are closed, and the degree of eye opening and closing.
7. Fatigue Judgment
8. The state of the eyes can most directly reflect the current driver's fatigue state. Commonly used eye states include blinking frequency, eye rotation frequency, and eye-closing duration. Among them, too low eyeball rotation frequency, too low eye blinking frequency, and long-term closed eyes can be regarded as fatigue.
9. Early Warning
10. That is, when the system determines that it is in a fatigue state, the buzzer sounds, or the system plays a piece of music to give an early warning.

RETRACTED

### 3.1. DCNN

The basic framework of DCNN is shown in Figure 1. It uses multilayer convolution and pooling to extract the high-level semantic features of the image. While ensuring the image rotation invariance and translation invariance, it reduces the dimension of the feature map and retains the important training process which is divided into two stages: forward propagation and back propagation [18]:

(1) *Forward-Propagation Stage*. The calculation process of the feature map input for each layer is
  (1) $$\begin{array}{c} Fe_{r}=f\left(\sum_{i\in I}w_{i}^{r}⊗x_{i}^{r-1}+e^{\beta_{i}^{r}}\right). \end{array}$$
Here, ⊗ represents the convolution operation, *Fe*_*r*_ represents the output of the *r-*th convolutional layer, *x*_*i*_^*r*−1^ is the input vector of the *r-*th layer, and *β*_*i*_^*r*^ is the bias term of the *r-*th layer; *I* is the set of input feature maps; *w*_*i*_^*r*^ is the weight of the *r-*th convolution kernel in the *r-*th layer; and *f*(∑_*i*∈*I*_*w*_*i*_^*r*^ ⊗ *x*_*i*_^*r*−1^+*β*_*i*_^*r*^) represents the activation function.
(2) *Back-Propagation Stage*. Assuming that the data set has *M* samples, the forward-propagation stage of the network will output the prediction results for each class, and the weights can be adjusted by comparing the expected output and the prediction results of the network [19]. Define the final objective function of the network as
  (2) $$\begin{array}{c} \mathrm{Exp}\left(W\right)=\text{Inf}\left\{\underset{M⟶\infty }{\lim}\sum_{i=1}^{M}\mathrm{Loss}\left(w_{i}\right)+\chi \left(w\right)\right\}. \end{array}$$

Here, Loss(*w*_*i*_) is the loss function, through iterative training to reduce the loss function of the network to reduce the classification error; *w*_*i*_ is the output of the last layer in formula (1), here representing the input of back propagation; *χ*(*w*) is the regular transformation function; and *w*_*i*_ represents the weight in the network.

### 3.2. Neural Network Parallel Optimization (NNPO) Algorithm

The NNPO algorithm mainly includes three stages: model compression, acquisition of local classification results, and acquisition of global classification results. (a) In the model compression stage, a feature map-based pruning strategy (PFM) is proposed to calculate the Loss() of the feature map. The norm gets the average value of the watt norm of the convolution kernel to realize the pruning of redundant parameters, pretrain the network, and obtain the compressed model. (b) In the phase of obtaining local classification results, first combine MapReduce parallel model and use split. The function divides the entire data set into file blocks of the same size, stores them on each node, and then uses the Map function to train the network on each node in parallel and proposes the conjugate gradient method (CGMSE) to modify the secant line to update the parameters, which improves the network convergence speed to obtain local classification results [20, 21]. In the stage of obtaining the global classification results, a load balancing strategy (LBRLA) is proposed to control the load rate to improve the parallelization performance of the parallel system. The Reduce function is used to obtain the final weight of the DCNN on each node to obtain the global classification result.

### 3.3. Model Compression

DCNN usually contains many layers, and each layer contains many convolution kernels. However, the weights in each convolution kernel are not helpful for network prediction, so the network contains a lot of redundant parameters. The usual redundant parameter pruning method is to calculate the *L*_*i*_ norm of each convolution kernel. Based on this, it is considered that the convolution kernel larger than the *L*_*i*_ norm is important, and the convolution kernel smaller than the *L*_*i*_ norm is not important. However, each convolution kernel actually represents a feature template at a specific level. For a shallower convolutional layer, as shown in Figure 2, the first convolutional layer of VGG16 can only extract simple edges [22]. Color blocks, for a deeper convolutional layer, are shown in Figure 2; the eighth conv4-VGG16 can concentrate on extracting highly abstract image features. Simply considering *L*, the norm may be wrong. Delete important convolution kernels, so this paper proposes a feature map-based pruning strategy (PFM) to pretrain DCNN before using all the data for training.

RETRACTED

The PFM strategy first randomly selects part of the training data to pretrain the DCNN and uses the average *L*_*i*_ norm of the output feature map of the convolution kernel to evaluate the importance of the convolution kernel. For each input sample *x* in the training data set, the *L*_*i*_ norm of the feature map *F* output by the convolution kernel can be calculated, followed by all the training samples. The mean value of the norm is assigned to the kernel, and the convolution kernel is sorted by the mean value of the *L*_*i*_ norm of the corresponding output feature map, and the convolution kernel whose mean value of the *L*_*i*_ norm is less than the preset threshold is prune to compress the model. This pruning strategy can repeat it to compress the model recursively and increase the calculation speed. The calculation formula of the *L*_*i*_ norm is

(3) $$\begin{array}{c} L_{i}=\underset{M⟶\infty }{\lim}\frac{\sum_{i=1}^{M}{\left(Fe_{i,j}-{\bar{Fe}}_{j}\right)}^{2}}{M^{2}}. \end{array}$$

Here, $Fe_{i,j}-{\bar{Fe}}_{j}$ represents the *L*_*i*_ norm of the feature map *Fe*_*i*,*j*_ corresponding to the output of the *j-*th convolution kernel when the *i-*th sample is input to the network; and *M* represents the number of samples randomly selected from the training data set.

### 3.4. Obtaining Local Classification

The acquisition of local classification results includes the split and map stages. In the split stage, the Hadoop default file block strategy is used to divide the original data into blocks of the same size; in the Map stage, the Map function is used to calculate the local change of each network weight parameter, update the weights, and obtain partial classification results. Since the stochastic gradient descent method of updating weights in the Map stage converges very slowly in the big data environment, based on the secondary convergence of the conjugate gradient method, this paper proposes a modified secant line of the conjugate gradient method (CGMSE) to find the optimal parameters and speed up the network convergence [23, 24].

RETRACTED

### 3.5. Obtaining Global Classification Results

Each node is trained to obtain the local weight of the DCNN, and MapReduce sends the key-value pair output by each Map node to the reduce() function to complete the final merge task to obtain the final network weight, where *w* is the weight, and (*a*, *b*) indicates that the weight is the *b*-th weight of the *a-*th convolution kernel. Considering the influence of load balancing on the efficiency of parallel algorithms, this paper proposes a load balancing strategy (LBRLA) to control the load rate. It can maintain the load balance of the parallel system through load distribution rules and set load thresholds and improve the utilization of system resources.

### 3.6. NNPO Algorithm Steps

The specific implementation steps of the NNPO algorithm are shown in Figure 3:

- In the model compression stage, according to the input original data set, pretrain the network by calling the PFM strategy of algorithm to perform model compression.
- In the phase of obtaining local classification results, first combine the MapReduce framework, call the split function to divide the data set, store it on each node, and then call the Map function to train the network on each node in parallel, and call the algorithm to perform parameter update to obtain partial classification results.
- In the phase of obtaining the global classification result, the LBRLA strategy of algorithm is called to control the load balancing of the parallel system, and the Reduce function is called to find the final weight of the network and obtain the final classification result [25].

## 4. Algorithm Experiment Results and Comparison

### 4.1. Experimental Data

At present, because the research work on fatigue detection and warning mainly stays at the level of automobile driving, relatively few are used for national security, but both have extremely high versatility in function, applicable objects, and applicable environment, so the research results and current status of fatigue detection and early warning of drivers largely represent the research results and current status of fatigue detection and early warning technology in the field of national security [26]. The experimental data used in this article are three real data sets, which are derived from Google data, namely, SV, E-digit, and ISL. In order to verify the time and space complexity of different algorithms, this paper conducts experiments based on the three data sets of SV, E-digit, and ISL and makes a comprehensive comparison based on the running time and memory usage. The SV data set contains color digital images from the real world, the size is 32 × 32, and there are 73,231 in the training set. There are 26,022 images and 531,312 images in the test set for additional training. No additional data is used this time. Instead, 6,000 images are segmented from the training set as the verification set, and the pixel value is divided by 255, so their size is in [0, 1); the E-digits data set is all 32 × 32 pixel black and white images. This data set provides a balanced handwritten digit data set that is directly compatible with the original data set. The training set is 240,000. The ISL data set contains 1,000 categories, 1,281,198 training images, 50,000 verification images, and 100,000 test images, each with more than 280,000 images in the test set. For two bounding boxes and corresponding class labels, the entire data set is about 150 GB, because the image size is not uniform, so the images in the data set are cropped and scaled to 224 × 224, and 500 of them are randomly selected for experiment.

RETRACTED

### 4.2. Evaluation Index

This article uses speedup as an indicator to evaluate the performance of the algorithm. The speedup of an algorithm refers to the performance improvement obtained through parallelization. It is usually used as an important indicator to test the performance of parallelized algorithms. The larger the speedup, the better the degree of parallelization of the algorithm. It is defined as

(4) $$\begin{array}{c} v=\frac{T_{s}}{T_{s}+T_{p}}. \end{array}$$

Here, *T*_*s*_ represents the serial execution time of the algorithm and *T*_*p*_ represents the parallel execution time of the algorithm.

### 4.3. Comparative Analysis of Algorithm Performance

In order to verify the time and space complexity of the NNPO algorithm, this paper conducts experiments based on the three data sets of SV, E-digit, and ISL. According to the running time and memory usage, it is compared with DCNN and the NNPO variants without network compression (hereinafter P-DCNN) for comprehensive comparison. Figures 4 and 5 show the execution time and memory usage of NNPO, MR-DCNN, and P-DCNN.

On the SV data set, the performance of NNPO is slightly better than those of MR-DCNN and P-DCNN. The execution times of MR-DCNN and P-DCNN are 33.15% and 21.24%, respectively. The memory usages of MR-DCNN and P-DCNN, respectively, are 55.71% and 56.16%; the execution time is less reduced because NNPO pretrains the network before classification, which affects the overall execution speed of the algorithm, and the memory usage is reduced more in the network after pruning. This is caused by the reduction in the number of redundant parameters. On the two larger data sets E-digit and ISL, the execution time and memory usage of the NNPO algorithm are much lower than those of MR-DCNN and P-DCNN. The running time of NNPO is 26.19% of that of MR-DCNN and P-DCNN, respectively. On the data sets E-digit and ISL, the memory usage of MR-DCNN and P-DCNN is 28.01%, 17.29%, 31.19%, and 17.92%, respectively. There are three reasons for this result: (a) Because the pretraining time is much smaller than the algorithm's execution time, it has little effect on the overall performance of the NNPO algorithm. (b) The conjugate gradient method using the modified secant line improves the network convergence speed, thereby reducing the execution time. (c) After the redundant parameters are pruned through the PFM strategy, the number of parameters is greatly reduced, and the program execution time and memory usage are also greatly reduced. On the whole, compare the running time and memory usage trend of NNPO, MR-DCNN, and P-DCNN on the three data sets. On the one hand, as the amount of data increases, the running time of NNPO increases less, while the running time of MR-DCNN increases more. The running times of P-DCNN and P-DCNN increase exponentially; on the other hand, the memory footprint of NNPO changes very little, while the memory footprints of MR-DCNN and P-DCNN increase sharply as the data set increases. Therefore, it can be concluded that NNPO is better than MR-DCNN and P-DCNN and can effectively improve the training efficiency of DCNN in a big data environment.

RETRACTED

After the algorithm NNPO in this paper prunes the redundant parameters through the PFM strategy, the number of parameters is greatly reduced, the sensitivity to the parameters is reduced, and the program execution time and memory usage are also greatly reduced.

## 5. Application of Algorithmic Exercise Fatigue Warning

The test of the system is carried out in a laboratory that simulates the on-duty environment of the on-duty personnel under real conditions. According to the actual usage, we limit the line of sight of the person to be inspected to 30 degrees up and down and within 30 degrees to the left and right, and the camera is placed at a distance of about 0.5 meters in front of the person to be monitored. The relevant parameters of the camera are set as follows: 640 × 480, 24 frames per second, with 1 minute as a test unit, and the collected image frames are 1440 frames. In the display window of the positioning results, use a red line to draw the human eye positioning results on the real-time video image frame; in the display window of real-time monitoring and early warning information, use waveform graphs to record that human eyes open and close over time, half-open and half-closed state value; what is displayed in the binarization window is the result of the image after binarization and its positioning result; what is displayed in the vertical projection window is the vertical projection result curve of the human eye area. For a single test time, calculate the PERCLOS value through the number of frames with human eyes closed and the total number of frames. If it is greater than 80%, an alarm will be issued. The test result and its success rate analysis are shown in Figures 6 and 7 .

RETRACTED

This automatic fatigue warning system uses a neural network parallel optimization algorithm based on big data to realize human eye positioning. After determining the human eye area, perform vertical integral projection operation on it, and determine the human eye state by calculating the characteristic parameter value of its projection curve; then calculate the PERCLOS value of the person to be tested in a period of time to achieve the purpose of judging the fatigue state. The relationship between PERCLOS value and fatigue is shown in Figure 8.

This method has the following advantages:

1. Human eye positioning is fast and accurate, and there is low false detection rate.
2. In terms of human eye positioning, the algorithm implements human eye positioning under the guidance of the main idea of “detecting human faces first and then detecting human eyes.” It not only inherits the characteristics of high detection success rate of face classifiers but also takes less time relatively. The search range of human eye positioning is narrowed, and the accuracy is correspondingly improved. At the same time, it greatly reduces the false alarm rate of the human eye classifier by removing false alarms on the algorithm.
3. The judgment of human eye condition is accurate, and there is high precision and simple process.
4. Compared with traditional algorithms for determining the state of the human eye, such as horizontal projection algorithms, the algorithm used in this system has a significant improvement in accuracy. The main difference is that it solves the accuracy problem of positioning the eyelid when judging the eye state by calculating the distance of the eyelid in the traditional algorithm. Traditional human eye state judgment algorithms often produce errors in judgment results due to the accuracy of positioning the eyelids and sometimes even unusable situations, but, in the test process of this system, such situations did not appear. The actual situation is basically the same. At the same time, it also showed some shortcomings of this system in some aspects, which needs to be improved in the future.
5. The interference of some external obstructions on target detection cannot be ruled out.
6. When the person to be monitored wears hats, glasses, bangs, masks, and so forth, which obscure facial features, the system eye positioning success rate will be greatly reduced. This is because when facial features are blocked, the system cannot obtain comprehensive and effective information. The first step of the human eye positioning algorithm will greatly reduce the success rate of face detection. If the face detection is unsuccessful, the following human eye positioning will naturally not be possible.
7. There are certain requirements for ambient light sources.
8. This system has certain requirements for the ambient light source, and the ambient light source must be within a certain range directly in front of the camera. If the ambient light source exceeds this range and exceeds the compensation capability of the illumination compensation in the image preprocessing, it will lead to the formation of a completely black face after the binarization, so that the human eye cannot be located.

RETRACTED

Tired work is one of the important causes of vicious accidents such as traffic accidents. Due to the fatigue of the staff working for a long time, such as inattention, frequent blinking, and too long time of closing the eyes, the response of the staff is slow, and accidents are easily caused. If a real-time detection system can be provided to give an alarm when people are first fatigued, accidents can be reduced and safety can be effectively improved.

## 6. Conclusion

The feature map-based pruning strategy (PFM) designed in this paper can effectively reduce redundant parameters and reduce the time and space complexity of DCNN training; and, in the subsequent Map stage, the fast convergence of the conjugate gradient method is realized, which improves the convergence speed of the network. In order to make up for the shortcomings of traditional DCNN in the big data environment, this paper proposes a new DCNN classification algorithm NNPO. First, randomly select part of the data for pretraining, and design a feature map-based pruning strategy (PFM), which reduces a large number of redundant parameters in DCNN by comparing the average value of the *L*_*i*_ norm of each convolution kernel, thereby reducing the time of the algorithm and space complexity; second, use MapReduce to conduct parallel training on DCNN, and propose a modified secant line conjugate gradient method (CGMSE) during the parameter update process of the Map stage, which is suitable for general situations and is improved by optimizing the search direction. The optimization efficiency is improved; finally, the load balancing strategy (LBRLA) to control the load rate is proposed in the Reduce stage, which solves the problem of unbalanced load of each node in the parallel system and improves the parallelization performance of the algorithm. Compared with the five algorithms of CNN-MR, the experimental results show that the speedup ratio of the NNPO algorithm is significantly higher than those of other algorithms in a big data environment. Finally, the algorithm is applied to the early warning system of fatigue detection. In the aspect of fatigue detection, the system uses the camera to take the image of the face of the person on duty. Then, according to the result of the human eye positioning, the vertical integral projection operation of the human eye area is performed to calculate the projection curve. The characteristic parameter value is used to determine the state of the human eye. Finally, according to the PERCLOS value of the person to be monitored for a certain period of time, it is judged whether they are in a fatigue state, and if they are fatigued, an early warning message is given.

RETRACTED

Fatigue feature extraction and fatigue determination are the core content of this article, but real-time fatigue warning is a very complex and challenging field. The fatigue early warning system studied in this paper is implemented in an ideal laboratory environment, but there are still many limitations in actual use. For example, in complex backgrounds such as fatigue warning of high-speed locomotives, rapid changes in the face and background, whether the user wears glasses or fatigue warning at night, and so forth are all tests of the system's real-time processing capabilities.

## Figures and Tables

**Figure 1:** DCNN structure.

**Figure 2:** Features of VGG16 output.

**Figure 3:** NNPO algorithm flow.

**Figure 4:** The execution time of the NNPO, MR-DCNN, and P-DCNN algorithms on the three data sets.

**Figure 5:** Memory usage of NNPO, MR-DCNN, and P-DCNN algorithms on three data sets.

**Figure 6:** The total number of frames with human eyes closed and opened.

**Figure 7:** Detection failure rate.

**Figure 8:** The relationship between PERCLOS value and fatigue.

## Data Availability

The data used to support the findings of this study are available from the corresponding author upon request.
